# Hsa_circ_0001944 promotes the growth and metastasis in bladder cancer cells by acting as a competitive endogenous RNA for miR-548

This article has been retracted.

**DOI:** 10.1186/s13046-020-01697-6

**Published:** 2020-09-14

**Authors:** Mingming Jin, Shengjie Lu, Yue Wu, Chen Yang, Chunzi Shi, Yanqiu Wang, Gang Huang

**Affiliations:** 1 Shanghai University of Traditional Chinese Medicine, Shanghai, 201203 PR China; 2 Shanghai Key Laboratory of Molecular Imaging, Shanghai University of Medicine and Health Sciences, 279 Zhouzhu Road, Pudong New Area, Shanghai, 201318 China; 3 Department of Urology, Huashan Hospital, Fudan University, Shanghai, China; 4 Reproductive medical center, Tongji Hospital, Tongji University School of Medicine, Shanghai, China

**Keywords:** Bladder cancer, hsa_circ_0001944, miR-548, PROK2, Proliferation

## Abstract

**Background:**

Bladder cancer (BC) is a common genitourinary malignancy worldwide. Circular RNAs (circRNAs) participate in cancer development, including BC; thus, the roles of circRNAs in this process have attracted significant attention.

**Methods:**

In this study, high-throughput sequencing was used to analyze circRNA expression profiles in BC tissues. We performed RT-qPCR to determine hsa_circ_0001944 expression in BC tissues. We used fluorescence in situ hybridization (FISH) to detect hsa_circ_0001944 expression and hsa_circ_0001944 subcellular localization in BC tissues. hsa_circ_0001944 expression in BC cells was selectively regulated. We employed CCK8, transwell, and wound healing assays to monitor cell proliferation, invasion, and migration, respectively. We employed the dual-luciferase reporter and RNA pulldown assays to verify the relationships among hsa_circ_0001944, miR-548, and PROK2. We examined the effects of hsa_circ_0001944 on BC cell metastasis and proliferation in vivo using a subcutaneous xenograft model and an intravenous tail injection model in nude mice.

**Results:**

The results showed that hsa_circ_0001944 expression was significantly increased in BC samples. Furthermore, high hsa_circ_0001944 expression predicted unfavorable prognoses in BC. Functional assays validated that downregulating hsa_circ_0001944 decreased BC invasion and proliferation in vivo and in vitro. Further studies showed that hsa_circ_0001944 expression promoted BC progression via sponging miR-548 and enhancing PROK2 expression. Luciferase reporter experiments validated the interactions between hsa_circ_0001944, miR-548, and PROK2. This study also found that downregulating miR-548 or overexpressing PROK2 restored BC cell invasion and proliferation after silencing hsa_circ_0001944.

**Conclusions:**

Taken together, we found that hsa_circ_0001944 is a tumor-promoting circRNA in BC that functions as a competing endogenous RNA to regulate PROK2 expression via sponging miR-548.

## Background

Globally, bladder cancer (BC) is the ninth most commonly diagnosed cancer in all patients and the fourth most frequent cancer diagnosis in men, with approximately 430,000 new BC patients diagnosed per year [1, 2]. Urothelial carcinoma (UC) is a transitional cell carcinoma that is a common BC subset. Currently, a definitive cure for UC is lacking, and its mortality rate has been relatively unchanged [3, 4]. In this regard, identifying new biomarkers and therapeutic targets for early BC diagnostics, especially UC, is an urgent public health demand .

Circular RNAs (circRNAs) belong to a family of single-stranded RNAs that construct a closed loop by joining their linear 5′ and 3′ ends [5, 6]. CircRNAs are ubiquitously expressed from archaea to eukaryotes and have highly evolutionary conserved functional roles. CircRNAs function as candidate biomarkers for the prognosis and diagnosis of cancer patients, and measuring circRNAs has been recommended by several investigations [7]. Studies have found that circ5912 suppresses cancer progression by inducing mesenchymal-to-epithelial transition in BC cells [8]. Circ-ITCH inhibits BC progression by sponging miR-17/miR-224 and regulating p21 and PTEN expression [9]. Studies have also found that hsa_circ_0001361 [10], circPICALM [11], hsa_circ_0137606 [12], and circ-ZKSCAN1 [13] function in BC progression. Although many circRNAs are known to have significant functions in cancer, more work is needed to confirm their impact on cancer genetics. Therefore, there is an urgent demand to identify more circRNAs and characterize their relevant molecular mechanisms in cancer.

This study found that hsa_circ_0001944 expression increased in BC tissues through high-throughput sequencing. We found that hsa_circ_0001944 expression predicted an unfavorable prognosis in BC patients. In vitro and in vivo experiments showed that hsa_circ_0001944 expression promoted BC invasion and proliferation by sponging miR-548 and enhancing PROK2 expression. Silencing hsa_circ_0001944 significantly suppressed BC invasion and proliferation. In summary, the data show that hsa_circ_0001944 is a tumor-promoting circRNA in BC by acting as competing endogenous (ce)RNA that regulates PROK2 expression through sponging miR-548. Finally, hsa_circ_0001944 should be treated as a candidate biomarker for detecting BC.

## Materials & methods

### Animals

We used 4-week-old BALB/c nude mice weighing 15–20 g (SLARC, Shanghai, China) in this study. The Ethics Committee of Shanghai University of Medicine and Health Sciences approved all animal experiments.

### Patients and samples

In total, we enrolled 90 pairs of BC tissues and adjacent normal tissues from BC patients who were treated at Huashan Hospital, Fudan University School of Medicine between January 2007 and January 2013. No patients received preoperative local or systemic treatment prior to specimen collection. We acquired informed consent from every patient or his/her relative(s). The Board and Ethics Committee of Huashan Hospital and Fudan University School of Medicine approved this project. We directly deposited collected tissues in liquid nitrogen for further usage.

### Strand-specific high-throughput RNA-Seq library construction

We extracted total RNA from paired BC and adjacent noncancerous tissues with TRIzol reagent (Invitrogen, Carlsbad, CA, USA). We subjected nearly 3 μg of total RNA from each sample to the VAHTS Total RNA-seq (H/M/R) Library Prep Kit from Illumina (Vazyme Biotech Co., Ltd., Nanjing, China) to erase ribosomal RNA, but retain other RNA classes such as non-coding RNAs and mRNAs. We treated the RNAs with 40 U of RNase R (Epicenter) at 37 °C for 3 h, followed by TRIzol purification. We prepared RNA-seq libraries by the KAPA Stranded RNA-Seq Library Prep Kit (Roche, Basel, Switzerland) and subjected them to deep sequencing through Illumina HiSeq 4000 at Aksomics, Inc. (Shanghai, China). For miRNA and mRNA analyses, T24 cells transfected with siRNA against hsa_circ_0001944 or negative control (NC) vector were used for high-throughput RNA-Seq of miRNAs as previously mentioned.

### Cell culture and transfection

We purchased SV-HUC-1 cells and the BC cell lines 5637, UM-UC-3, T24, and RT-4 from Type Culture Collection in Chinese Academy of Sciences (Shanghai, China) and cultured them in DMEM (Gibco, Grand Island, NY, USA) supplemented with 10% fetal bovine serum (FBS) at 37 °C in a humidified incubator with 5% CO_2_.

We transfected small interfering RNAs (siRNAs; si-hsa_circ_0001944 and si-circRNA), miR-548 mimics, miR-548 inhibitors, PROK2 overexpression vector, and their NCs into cultured T24 or UM-UC-3 cells via Lipofectamine 2000 (Invitrogen, Carlsbad, CA, USA) following the standard process. To further verify the effect of hsa_circ_0001944 using in vivo experiments, lentiviral-stabilized hsa_circ_0001944-silenced (sh-circ0001944) T24 cells were constructed.

### Bioinformatic analysis

We identified circRNA/miRNA target genes with *CircularRNAInteractome*. We predicted the interactive relationship between miR-548 and PROK2 using *TargetScanHuman*.

### Fluorescence in situ hybridization (FISH)

We made specific probes against hsa_circ_0001944 (Dig-5′-GATACTTTATGAGGAGACTAAGGTGTCAGTATG-3′-Dig) with help from Geneseed Biotech (Guangzhou, China). We explored signals using Cy3-conjugated anti-digoxin and FITC-conjugated anti-biotin antibodies (Jackson ImmunoResearch Inc., West Grove, PA, USA). We counterstained nuclei with 4,6-diamidino-2-phenylindole (DAPI). Afterwards, we acquired images with a Zeiss LSM 700 confocal microscope (Carl Zeiss, Oberkochen, Germany).

### Total RNA isolation and quantitative reverse transcription (RT-q)PCR

We isolated total RNA from tumor tissues or cells with TRIzol reagent (Invitrogen) following the standard protocol. We examined RNA samples for purity and concentration spectrophotometrically by detecting absorbance at 260 nm, 280 nm, and 230 nm with a NanoDrop ND-1000 (Thermo Fisher Scientific, Wilmington, DE, USA). In particular, we deemed OD260/OD280 ratios ranging between 1.8–2.1 and OD260/OD230 ratios > 1.8 as acceptable.

We reverse transcribed total RNA before RT-qPCR detection. We obtained primers specific for hsa_circ_0001944, miR-548, and PROK2 from GenePharma (Shanghai, China). We performed RT-qPCR with AB7300 thermo-recycler (Applied Biosystems, Carlsbad, CA, USA) with primers and the TaqMan Universal PCR Master Mix. We employed *GAPDH* as reference gene for circRNAs and mRNAs. We used U6 as an internal control for miRNA expression levels. We quantified gene expression via the 2^−ΔΔCt^ method. The primers utilized to assay *hsa_circ_0001944* expression included 5′-CTCTTTGACATCATAATAAAATACT-3′ forward, and 5′-GGCTGAGGCAGGAGAATAGCTTGGG-3′ reverse. The *miR-548* primers were 5′-ATTGGAACGATACAGAGAAGATT-3′ forward and 5′-GGAACGCTTCACGAATTTG-3′ reverse. The *PROK2* primers were 5′-GGGGATCCATGAGGAGCCTGTGCTGCGCCCCA-3′ forward, and 5′-GGGAATTCCTTTTGGGCTAAACAAATAAATCG-3′ reverse. The *U6* primers were 5′-CTCGCTTCGGCAGCACA-3′ forward, and 5′-AACGCTTCACGAATTTGCGT-3′ reverse. The *GAPDH* primers were 5′-GCACCGTCAAGGCTGAGAAC-3′ forward, and 5′-GGATCTCGCTCCTGGAAGATG-3′ reverse.

### Dual-luciferase reporter assays

We inserted binding sites for hsa_circ_0001944 and the PROK2 3′-UTR, termed hsa_circ_0001944-WT, hsa_circ_0001944-Mut, PROK2–3′UTR-WT, and PROK2–3′UTR-Mut into HindIII and KpnI sites of pGL3 promoter vector (Realgene, Nanjing, China) of the dual-luciferase reporter assay. We first plated cells into 24-well plates, and transfected 80 ng of plasmid, 50 nM of miR-548 mimics, 5 ng of the Renilla luciferase vector pRL-SV40, and NC reagents into cells with lipofectamine 2000 (Invitrogen). We collected cells and measured them 2 d after transfection with Dual-Luciferase Assay (Promega, Madison, WI, USA), following standard instructions. We independently repeated all experiments three times.

### Cell proliferation assay

We used the Cell Counting Kit-8 (CCK-8) assay to detect cell proliferation. We seeded transfected cells into 96-well plates at a density of 5000 cells/well in triplicate. We measured cell viability through the CCK-8 system (Gibco) at 0, 1, 2, and 3 d after seeding, following standard procedures.

For colony formation assays, we seeded transfected cells into six-well plates at a density of 2000 cells/well and maintained them in DMEM containing 10% FBS for 10 d. We imaged and counted the resultant colonies after fixing and staining them.

### 5-Ethynyl-2′-deoxyuridine (EdU) assay

We used the EdU assay kit (RiboBio, Guangzhou, China) to investigate cell proliferation and DNA synthesis. We seeded 10,000 T24 or UMUC3 treated cells into 96-well plates overnight. The second day, we added EdU solution (25 μM) to the plate and incubated the cells for 1 d. We then used 4% formalin to fix the cells at room temperature for 2 h. We utilized 0.5% TritonX-100 to permeabilize the cells for 10 min, and added Apollo reaction solution (200 μL) to stain EdU and DAPI (200 μL) to stain nuclei for 30 min. Lastly, a Nikon microscope (Nikon, Tokyo, Japan) was used to measure cell proliferation and DNA synthesis, which were reflected by blue and red signals, respectively.

### Transwell and wound healing assays

We suspended BC cells in 200 μL of serum-free medium and inserted them into upper chamber of Transwell plates with 8-μm pores (Corning Costar, Corning, NY, USA). We also placed 600 μL medium containing 20% FBS in lower chamber as chemoattractant. After incubation for 1 d, we fixed cells in the filter with methanol, stained them with 0.1% crystal violet solution, and then counted them in three random fields of view (200×).

For wound healing assays, we seeded BC cells in 6-well plates. We created a linear scratch wound with a 20-μL pipette tip in the confluent monolayer of cells. After 2 d of incubation in medium without FBS, we observed and photographed wound closure under microscope. We conducted experiments in triplicate and repeated them three times.

### Flow cytometric analysis of cell cycle progression

We fixed cells in 70% ethanol overnight at 4 °C, resuspended them in staining solution (Beyotime, Shanghai, China), and then incubated them for 30 min at 4 °C. We measured stained cells by flow cytometry (Beckman Coulter, Franklin Lakes, NJ, USA).

### Animal studies

For the xenograft assays, we subcutaneously injected 1 × 10^6^ modified (hsa_circ_0001944-silenced) or NC T24 cells into the right side of each male nude mouse. We calculated tumor volumes (length × width^2^ × 0.5) at the indicated timepoints and excised tumors 4 weeks after the injection.

For metastasis analysis, we transfected 2 × 10^5^ NC or hsa_circ_0001944-silenced T24 cells with luciferase expression vectors, and injected the cells intravenously into the tails of mice. After 30 d, T24 cell metastases were analyzed by bioluminescence imaging following an intravenous injection of luciferin (150 mg luciferin/kg body weight) into the tails.

### Immunohistochemistry

We fixed tumor tissue samples in 10% formalin and embedded them in paraffin. We stained sections (5-μm thick) with Ki67 to explore proliferation. We examined sections with an Axiophot light microscope and imaged them with digital camera.

### Statistical analysis

We assessed differences among groups via paired/unpaired *t*-tests (two-tailed). We used Pearson’s correlation test to obtain associations between groups. Data are presented as mean ± SEM. We considered *P*-values < 0.05 as significant. We performed all statistical analyses with GraphPad Prism (GraphPad Inc., San Diego, CA, USA).

## Results

### High hsa_circ_0001944 expression predicted unfavorable prognoses for BC patients

To reveal correlations between circRNA expression and BC progression, two BC samples were used for circRNA high-throughput sequencing. The results show that 2113 circRNAs were upregulated and 1551 circRNAs were downregulated in BC tissues compared with adjacent normal tissues (Fig. 1a). However, only 12 circRNAs were significantly upregulated and 78 were significantly downregulated (Fig. 1b). Among the upregulated circRNAs, hsa_circ_0001944 expression was significantly increased in BC tissues (supplementary materials. S1). FISH assays demonstrated that hsa_circ_0001944 expression increased in BC tissues compared with adjacent normal tissues. The results also showed that hsa_circ_0001944 was localized predominately to cytoplasm (Fig. 1d). RT-qPCR detection of 90 patient samples suggested hsa_circ_0001944 expression increased in BC tissues compared with adjacent normal tissues (Fig. 1e). To further understand prognostic value of hsa_circ_0001944 expression, we analyzed correlations with patient characteristics. This illustrated that high hsa_circ_0001944 expression was correlated with increased tumor size, higher stage, lymph node metastasis, and higher pathological T stage (Table. 1). Also, the correlation analysis demonstrated that high hsa_circ_0001944 expression was associated with poorer overall survival compared with patients with low hsa_circ_0001944 expression (Fig. 1f). hsa_circ_0001944 is derived from circularizing exons from gene *TCONS_l2_00030860*, which located at chr5:73069679–73,076,570. *TCONS_l2_00030860* consists of 45,161 bp and spliced mature circRNA is 1096 bp (Fig. 1g). In this regard, these findings suggest that hsa_circ_0001944 functions in BC progression.

**Fig. 1:** High hsa_circ_0001944 expression predicted an unfavorable prognosis in BC patients. **a** The total differential expression of circRNAs. **b** Volcano plots illustrate that among significantly different expressed circRNAs, 12 were upregulated and 78 were downregulated in BC tissues relative to normal tissues. **c** The expression and subcellular localization of hsa_circ_0001944 in BC was analyzed by in situ hybridization in a BC tissue. **d** RT-qPCR detection show the differential expression of hsa_circ_0001944 in 90 paired BC tissues. Data are presented as mean ± SD; ^***^P < 0.001 vs. normal group. **e** hsa_circ_0001944 expression among 90 patients was analyzed for overall survival. **f** The genomic locus of hsa_circ_0001944

**Table 1:** Relationship between the expression levels of hsa_circ_0001944 and clinicopathological features in bladder cancer

Characteristics	No. (%)	hsa_circ_0001944 expression		
		Low (%)	High (%)	*P*-value
**Gender**				
Male	42 (46.7)	23 (54.8)	19 (45.2)	0.347
Female	48 (53.3)	29 (60.4)	19 (39.6)	
**Age**				
< 65	38 (42.2)	20 (52.6)	18 (47.4)	0.186
≥ 65	52 (57.8)	32 (61.5)	20 (38.5)	
**Tumour size**				
< 3 cm	55 (61.1)	40 (72.7)	15 (27.3)	0.031
≥ 3 cm	35 (38.9)	12 (34.3)	23 (65.7)	
**Pathology stage**				
pTa-pT1	57 (63.3)	43 (75.3)	14 (24.7)	0.012
pT2-T4	33 (36.7)	9 (27.3)	24 (72.7)	
**Grade**				
Low	58 (64.4)	41 (70.7)	17 (29.3)	0.014
High	32 (35.6)	11 (34.4)	21 (65.6)	
**Lymphatic metastasis**				
Yes	19 (21.1)	5 (26.3)	14 (73.7)	0.017
No	71 (78.9)	47 (66.2)	24 (33.8)	
Total	90	52	38	

### Silencing hsa_circ_0001944 suppressed BC proliferation in vivo and in vitro

Rt-qPCR experiments showed that hsa_circ_0001944 expression in BC cell lines was increased compared with the normal cell line SV-HUC-1 (Fig. 2a). T24 and UMUC3 cells had the highest hsa_circ_0001944 levels, so they were selected for further experiments. hsa_circ_0001944 expression was significantly decreased in both UMUC3 and T24 cells after transfecting a siRNA against hsa_circ_0001944 (Fig. 2b). Cell cycle distribution analysis demonstrated that the S-phase proportion was significantly decreased, while the G2/M-phase proportion was increased after hsa_circ_0001944 depletion (Fig. 2c), suggesting a cell cycle arrest at G2/M phase. CCK8 (Fig. 2d and e), colony formation assays (Fig. 2f and g), and DNA synthesis determination by the EdU assay (Fig. 2h and i) showed that silencing hsa_circ_0001944 suppressed cell proliferation in UMUC-3 and T24 cells. The xenograft results verified that hsa_circ_0001944 knockdown suppressed T24 tumor growth (both weight and volume) compared with the NC group (Fig. 3a-c). Immunohistochemical detection of Ki67 demonstrated that hsa_circ_0001944 silencing suppressed Ki67 expression in tumor tissues (Fig. 3d), which verified that hsa_circ_0001944 knockdown suppressed tumor growth. RT-qPCR analysis showed that silencing hsa_circ_000194 decreased hsa_circ_000194 and PROK2 expression in tumor tissues, but promoted miR-548 expression (Fig. 3e-g).

**Fig. 2:** Downregulation of hsa_circ_0001944 suppressed BC proliferation in vitro. **a** RT-qPCR detection showing the expression of hsa_circ_0001944 in different BC cell lines. Data are presented as mean ± SD; ^***^P < 0.001 vs. the SV-HUC-1 group. **b** RT-qPCR detection showing the expression of hsa_circ_0001944 in both T24 and UMUC3 cells after transfection with siRNA against hsa_circ_0001944 or negative control. Data are presented as mean ± SD; ^***^P < 0.001 vs. the NC. **c** Flow cytometry detection showing the percentages of cells in G1, S, or G2 phase in both T24 (C) and UMUC3 (D) cells. **d** and **e** CCK8 assays were used to evaluate cell proliferation. Data are presented as mean ± SD; ^***^P < 0.001 vs. NC. **f** and **g** Colony formation assay showing proliferation in both T24 and UMUC3 cells. Data are presented as mean ± SD; ^***^P < 0.001 vs. NC. **h** and **i** Edu assays were used to evaluate cell proliferation. Data are presented as mean ± SD; ^***^P < 0.001 vs. NC

**Fig. 3:** Xenograft tumor studies. **a**-**c** T24 cells transfected with NC or sh-circ0001944 were subcutaneously injected into nude mice, and tumor growth curves and tumor weight were plotted. Data are presented as mean ± SD; **P < 0.01, ***P < 0.001 vs. NC. **d** Immunohistochemistry showing the percentage of Ki-67-positive cells. **e**-**g** RT-qPCR detection show the expression of hsa_circ_0001944 (E), miR-548 (F) and PROK2 (G) in tumor tissues. Data are presented as mean ± SD; ^***^P < 0.001 vs. NC

### Silencing hsa_circ_0001944 suppressed BC invasion in vitro and in vivo

Transwell migration (Fig. 4a and b) and wound healing (Fig. 4c and d) assays to detect for invasive ability showed that silencing hsa_circ_0001944 decreased migration and invasion of both T24 and UMUC-3 cells. The metastasis ability of T24 cells was also decreased after hsa_circ_0001944 silencing using live imaging analysis of metastasis model mice (Fig. 4e). Together, these data suggest that knocking down hsa_circ_0001944 suppressed the invasion ability of BC cells both in vivo and in vitro*.* Immunohistochemical detection of Ki67 demonstrated that hsa_circ_0001944 silencing suppressed Ki67 expression in metastatic lung tissue (Fig. 3f), which verified that hsa_circ_0001944 knockdown suppressed tumor growth. RT-qPCR analysis showed that silencing hsa_circ_000194 decreased hsa_circ_000194 and PROK2 expression in metastatic lung tissue, but promoted miR-548 expression (Fig. 3g-i).

**Fig. 4:** Downregulation of hsa_circ_0001944 suppressed BC invasion both in vitro and in vivo. **a** and **b** Cell migration was assessed in both T24 and UMUC3 cells using transwell assays. Data are presented as mean ± SD; ^***^P < 0.001 vs NC. **c** and **d** Wound healing assays show the invasion ability of both T24 and UMUC3 cells. Data are presented as mean ± SD; ^***^P < 0.001 vs NC. **e** Live imaging showing the effects of hsa_circ_0001944 on the metastasis of T24 cells 30 d after intravenous tail injection. **f** Immunohistochemistry showing the percentage of Ki-67-positive cells. **g**-**i** RT-qPCR detection show the expression of hsa_circ_0001944 (G), miR-548 (H) and PROK2 (I) in tumor tissues. Data are presented as mean ± SD; ^***^P < 0.001 vs. NC

### miR-548 and PROK2 are relevant downstream targets of hsa_circ_0001944 in BC

Increasingly, studies have confirmed that circRNAs, including microRNA (miRNA/miR) response elements, interact with miRNAs as competitive endogenous RNAs (ceRNAs) to regulate target mRNA expression [14, 15]. Therefore, we selected T24 cells with or without hsa_circ_0001944 silencing for high-throughput sequencing. The results showed that hsa_circ_0001944 depletion resulted in a series of upregulated miRNAs (supplementary materials. S2). Combined with the biological analysis that showed miR-548 was a hsa_circ_0001944 target, bioinformatic analyses also illustrated that miR-548 was a downstream hsa_circ_0001944 target (Fig. 5a). To further verify the relationship between hsa_circ_0001944 and miR-548, we prepared wild-type (WT) or mutated (MUT) hsa_circ_0001944 sequences that included the miR-548 binding sequence into a luciferase reporter vector (Fig. 5b). We then transfected this reporter vector into 293 T cells combined with a miR-548 mimic or not. Luciferase reporter analysis suggested that miR-548 inhibited luciferase activity in WT-transfected cells, yet not in MUT-transfected cells (Fig. 5c), suggesting that miR-548 was a hsa_circ_0001944 target.

**Fig. 5:** miR-548 and PROK2 are downstream targets of hsa_circ_0001944. **a** Venn diagram from Interactome (https://circinteractome.nia.nih.gov/), and high-throughput sequencing of miRNAs predicted to be sponged by hsa_circ_0001944. **b** Bioinformatics analysis prediction of binding sites of miR-548 in hsa_circ_0001944. The mutant version of hsa_circ_0001944 is presented. **c** Relative luciferase activity determined 48 h after transfecting HEK293T cells with miR-548 mimic/NC or hsa_circ_0001944 wild-type/Mut. Data are presented as means ± SD. ***P < 0.001. **d** Prediction of binding sites of miR-548 within the 3′-UTR of PROK2. The mutant version of the 3′-UTR-PROK2 is shown. **e** Relative luciferase activity 48 h after transfecting HEK293T cells with miR-548 mimic/NC or 3′-UTR-PROK2 wild-type/Mut. Data are presented as means ± SD. ***P < 0.001. **f**-**k** RT-qPCR detection show the expression of hsa_circ_0001944 (F and G), miR-548 (H and I), and PROK2 (J and K) in both T24 and UMUC3 cells. Data are presented as means ± SD. *P < 0.05, ***P < 0.001 vs NC. ^##^*P* < 0.01, ^###^*P* < 0.001 vs si-circRNA

Bioinformatic analyses illustrated that PROK2 was a miR-548 downstream target. To further validate the correlation between miR-548 and PROK2, we constructed WT or MUT 3′UTR-PROK2 sequences that included that miR-548 binding sequence into a luciferase reporter vector (Fig. 5d). We then transfected this reporter vector into 293 T cells combined with a miR-548 mimic or not. Luciferase reporter analysis demonstrated that miR-548 inhibited luciferase activity in WT-transfected cells, yet not in MUT-transfected cells (Fig. 5e), suggesting that PROK2 was a miR-548 target.

To identify the regulatory relationships between hsa_circ_0001944, miR-548, and PROK2, both T24 and UMUC3 cells were transfected with si-hsa_circ_0001944, miR-548 inhibitor or PROK2 overexpression vector, either singly or in combination. RT-qPCR detection showed that hsa_circ_0001944 expression decreased significantly after transfection with the siRNA against hsa_circ_0001944. miR-548 downregulation or PROK2 overexpression could not reverse the hsa_circ_0001944 expression in UMUC3 or T24 cells (Fig. 5f and h). hsa_circ_0001944 downregulation increased miR-548 expression in UMUC3 and T24 cells. Treating cells with the miR-548 inhibitor suppressed miR-548 expression, but PROK2 overexpression could not reverse miR-548 expression (Fig. 5j and g). We also found that silencing hsa_circ_0001944 decreased PROK2 expression in both T24 and UMUC3 cells, while treatment with the miR-548 inhibitor partially recovered PROK2 expression. Transfecting the PROK2 overexpression vector increased PROK2 expression (Fig. 5i and k). Together, these data suggest that miR-548 and PROK2 are downstream targets of hsa_circ_0001944 and that PROK2 is a miR-548 downstream target.

### Silencing miR-548 or overexpressing PROK2 restored invasion and proliferation of BC cells after removing hsa_circ_0001944

Colony formation (Fig. 6a-c) and EdU (Fig. 6d-f) assays showed that silencing hsa_circ_0001944 suppressed the proliferation of both UMUC3 and T24 cells. Further silencing miR-548 or overexpressing PROK2 rescued proliferation ability of UMUC3 and T24 cells. Transwell assays to measure cell invasion (Fig. 6g-i) also found that silencing miR-548 or overexpressing PROK2 rescued invasion ability of both T24 and UMUC3 cells.

**Fig. 6:** Downregulation miR-548 or overexpression PROK2 restored the proliferation and invasiveness of BC cells after has_circ_0001944 was silenced. **a**-**c** Colony formation assays show the proliferation of both T24 and UMUC3 cells after transfection with si-hsa_circ_0001944, miR-548 inhibitor, or PROK2 overexpression vector, either singly or in combination. Data are means ± SD. ***P < 0.001 vs. NC. ^###^*P* < 0.001 vs. si-circRNA. **d**-**f** Edu assay shows the proliferation of both T24 and UMUC3 cells after transfection with si-has_circ_0001944, miR-548 inhibitor, or PROK2 overexpression vector, either singly or in combination. Data are means ± SD. ***P < 0.001 vs. NC. ^###^*P* < 0.001 vs. si-circRNA. **g**-**i** Transwell migration assays of both T24 and UMUC3 cells. Data are means ± SD. ***P < 0.001 vs. NC. ^###^*P* < 0.001 vs. si-circRNA

### Overexpressing PROK2 restored invasion and proliferation of BC cells after overexpressing miR-548

Colony formation (Fig. 7a-c) and EdU (Fig. 7d-f) assays showed that overexpressing miR-548 suppressed proliferation of T24 and UMUC3 cells. Overexpressing PROK2 rescued the proliferation ability of T24 and UMUC3 cells because miR-548 could not interact with exogenous PROK2, which lacked a 3′UTR after transcription. Transwell assays to measure cell invasion (Fig. 7g-i) also found that overexpressing PROK2 rescued the invasion ability of both T24 and UMUC3 cells that overexpressed miR-548.

**Fig. 7:** PROK2 overexpression rescued the proliferation and invasiveness of BC cells after miR-548 upregulation. **a**-**c** Colony formation assays show the proliferation of both T24 and UMUC3 cells after transfection with miR-548 mimic or PROK2 overexpression vector, either singly or in combination. Data are means ± SD. ***P < 0.001 vs. NC. ^###^*P* < 0.001 vs. si-circRNA. **d**-**f** Edu assays show the proliferation of both T24 and UMUC3 cells after transfection with si-hsa_circ_0001944, hsa_circ_0001944 inhibitor, or PROK2 overexpression vector, either singly or in combination. Data are means ± SD. ***P < 0.001 vs. NC. ^###^*P* < 0.001 vs. si-circRNA. (G-I) Transwell migration assays of both T24 and UMUC3 cells. Data are means ± SD. ***P < 0.001 vs. NC. ^###^*P* < 0.001 vs. si-circRNA

## Discussion

CircRNAs belong to a new class of ncRNAs that have attracted significant research attention, as they may have important functions in gene expression and signaling pathways that participate in disease processes. As previously mentioned, circRNAs have tremendous potential for diagnosing tumors. Our high-throughput sequencing study found that hsa_circ_0001944 expression increased in BC tissues. Our clinical study verified that hsa_circ_0001944 expression correlated with lymph node metastasis, increased tumor size, higher stage, and higher pathological T stage. We also found that high hsa_circ_0001944 expression correlated to poorer overall survival. Thus, these findings suggest that hsa_circ_0001944 plays a role in BC progression.

This study also found that hsa_circ_0001944 expression was increased in BC cell lines. Silencing hsa_circ_0001944 suppressed cell invasion and proliferation in vitro and in vivo. The role of non-coding circRNAs as miRNA “sponges” has been previously demonstrated [16, 17]. Our bioinformatic analyses and high-throughput sequencing verified that miR-548 was a hsa_circ_0001944 target, which was confirmed by luciferase reporter assays.

Previous studies have found that miR-548 was significantly downregulated in prostate cancer tissues and correlated with advanced TNM stage, increased tumor size, distant metastasis, and poor prognosis. Additionally, miR-548 overexpression significantly inhibited prostate cancer cell invasion and proliferation in vivo and in vitro [18]. Other studies have found that miR-548 expression can suppress the progression of breast cancer [19] and hepatocellular carcinoma [20]. This study found that miR-548 expression suppressed the invasion and proliferation of BC cells. Silencing miR-548 rescued the invasion and proliferation abilities of UMUC3 and T24 cells after hsa_circ_0001944 was silenced. Therefore, the findings suggest that hsa_circ_0001944 promotes BC progression by sponging miR-548.

Previous studies have found that miR-548 can interact with the 3′UTR of Prokineticin 2 (PROK2) and suppress its expression. PROK2 is a cysteine-rich secreted protein that is expressed in testis and at lower levels in small intestine. PROK2 belongs to the prokineticin protein family, which have a conserved AVITGA and 10 cysteines in their N-terminal sequence. The gene encoding PROK2 is located on chromosome 3p21.1, which associates with the progress of malignant tumors [21–23]. Studies have found that PROK2 overexpression increases cancer cell proliferation and invasion, including in colorectal cancer [24], prostate cancer [25], breast cancer [26], and hepatocellular carcinoma [27]. Our study found that silencing hsa_circ_0001944 decreased PROK2 expression by enhancing miR-548 expression. Exogenously overexpressing PROK2 rescued the invasion and proliferation abilities of T24 and UMUC3 cells after silencing hsa_circ_0001944 silence or upregulating miR-548. These findings suggest that hsa_circ_0001944 promotes BC progression via sponging miR-548, which enhances PROK2 expression.

## Conclusion

In summary, these data illustrated that hsa_circ_0001944 expression increased in BC and was closely correlated to BC development and occurrence. We showed that hsa_circ_0001944 directly targets miR-548, which leads to increased PROK2 expression. Silencing hsa_circ_0001944 suppressed BC progression by increasing miR-548 levels, which led to decreased PROK2 expression. Thus, our findings provide a novel target for BC treatment that warrants further investigation.

## Supplementary information

**Additional file 1.**

## Data Availability

The data generated or analyzed during this study are included in this article, or if absent are available from the corresponding author upon reasonable request.

## Abbreviations

BC: Bladder cancer
circRNAs: Circular RNAs
FISH: Fluorescence in situ hybridization
PROK2: Prokineticin 2
CCK-8: Cell Counting Kit-8
DAPI: 4,6-diamidino-2-phenylindole
miRNA: MicroRNA
ceRNAs: Competitive endogenous RNAs
WT: Wild-type
MUT: Mutated
